# Circular RNA circ_0003204 inhibits proliferation, migration and tube formation of endothelial cell in atherosclerosis via miR-370-3p/TGFβR2/phosph-SMAD3 axis

**DOI:** 10.1186/s12929-019-0595-9

**Published:** 2020-01-03

**Authors:** Shanchao Zhang, Guixiang Song, Jing Yuan, Shan Qiao, Shan Xu, Zhihua Si, Yang Yang, Xuxu Xu, Aihua Wang

**Affiliations:** Department of Neurology, the First Affiliated Hospital of Shandong, First Medical University, NO.16766 JingShi Road, Jinan, 250014 Shandong China

**Keywords:** Hsa_circ_0003204, MiR-370-3p, TGFβR2, Endothelial cell, Atherosclerosis

## Abstract

**Background:**

Circular RNAs (circRNAs) represent a class of non-coding RNAs (ncRNAs) which are widely expressed in mammals and tissue-specific, of which some could act as critical regulators in the atherogenesis of cerebrovascular disease. However, the underlying mechanisms by which circRNA regulates the ectopic phenotype of endothelial cells (ECs) in atherosclerosis remain largely elusive.

**Methods:**

CCK-8, transwell, wound healing and Matrigel assays were used to assess cell viability, migration and tube formation. QRT-qPCR and Immunoblotting were used to examine targeted gene expression in different groups. The binding sites of miR-370-3p (miR-370) with TGFβR2 or hsa_circ_0003204 (circ_0003204) were predicted using a series of bioinformatic tools, and validated using dual luciferase assay and RNA immunoprecipitation (RIP) assay. The localization of circ_0003204 and miR-370 in ECs were investigated by fluorescence in situ hybridization (FISH). Gene function and pathways were enriched through Metascape and gene set enrichment analysis (GSEA). The association of circ_0003204 and miR-370 in extracellular vesicles (EVs) with clinical characteristics of patients were investigated using multiple statistical analysis.

**Results:**

Circ_0003204, mainly located in the cytoplasm of human aorta endothelial cells (HAECs), was upregulated in the ox-LDL-induced HAECs. Functionally, the ectopic expression of circ_0003204 inhibited proliferation, migration and tube formation of HAECs exposed to ox-LDL. Mechanically, circ_0003204 could promote protein expression of TGFβR2 and its downstream phosph-SMAD3 through sponging miR-370, and miR-370 targeted the 3′ untranslated region (UTR) of TGFβR2. Furthermore, the expression of circ_0003204 in plasma EVs was upregulated in the patients with cerebral atherosclerosis, and represented a potential biomarker for diangnosis and prognosis of cerebrovascular atherogenesis.

**Conclusions:**

Circ_0003204 could act as a novel stimulator for ectopic endothelial inactivation in atherosclerosis and a potential biomarker for cerebral atherosclerosis.

## Introduction

Atherosclerosis, characterized as lipid deposition and fibrous cap formation in the arterial wall, is a chronic inflammatory disease that contributes to most common vascular diseases, such as cerebral infarction, cardiovascular disease, which give rise to high mortality in aged population [1–3]. Aberrant ECs injury is regarded as one of pathological characteristics in the progression of atherosclerosis [4]. During the initiation and development of atherosclerosis, ECs are exposed to various pathogenic threats, such as ox-LDL, which display abnormal proliferation, migration and vasculogenesis that are responsible for breakdown of the integrity of endothelium to aggravate lipid deposition and fibrous cap rupture in return [5, 6]. Besides, damaged ECs produce multiple types of cytokines which refer to interleukin, adhesion molecules, matrix metalloproteinases, etc., which participate in the atherogenesis [7]. Therefore, the study on the unknown molecular mechanisms underlying EC aberrant transformation in atherosclerosis could provide us with potential targets for reversing EC injury and clinical prevention.

Overwhelming evidences have indicated that variable microRNA alterations are associated with atherosclerotic plaque progression and regression [8, 9]. For example, the expression of miR-103 is significantly upregulated in ox-LDL-exposed HAECs, and miR-103 directly blocks PTEN expression for activating MAPK signaling pathway, which are involved in inflammation process and endoplasmic reticulum stress in atherosclerosis plaque [10]. Importantly, in addition to miRNA, other ncRNAs, such as long intergenic ncRNAs and circRNAs also are involved in pathological process of atherosclerosis [11, 12]. Noticeably, circRNAs, formed by non-sequential back-splicing of pre-mRNA transcript, are widely expressed in eukaryotic cells and characterized by tissue-specific expression [13]. Compared with linear RNAs, circRNAs have characteristic stable structure of covalently closed loops without a free 5′ or 3′ end [14]. These traits strongly imply that circRNAs might serve as potential biomarkers for human disease. Recently, growing evidences indicated circRNAs may participate in the atherogenesis in the way as interaction with RNA-binding protein (RBP) or miRNA sponges to alter downstream gene expressions [11, 15], for example, previous data have suggested that the circANRIL modulates ribosomal RNA maturation through binding with pescadillo homologue 1, which, as a consequence, induces cellular proliferation inhibition and apoptosis in atherosclerosis plaque [11]. Additionally, aberrant upregulation of circCHFR in the ox-LDL-induced vascular smooth muscle cell (VSMCs) enhances the proliferation and migration of VSMCs by sponging miR-370, leading to vascular remodeling and the generation of collagen fibers [16]. However, little is known about the functional role of circRNAs in EC aberrant phenotype in atherosclerosis. A recent study reported that increased expression of circ_0003575 by ox-LDL could block the proliferation and angiogenic ability of human umbilical vein endothelial cell (HUVEC) [17]. Although this previous study never explored the detailed mechanisms upon circRNA function underlying EC injury in depth, it provides a hypothesis that circRNAs may act as crucial regulator of aberrant EC phenotype in the atherogenesis, which, hence, is the focus of our present study.

In the current study, we identified a circRNA (circ_0003204) in HAECs, and further investigated its expression and function by in vitro model and expressive profile in the plasma EVs from the patients with cerebral atherosclerosis. We found that circ_0003204 may act as a competing endogenous RNA (ceRNA) to regulate TGFβR2 and its downstream gene by decoying the miR-370, leading to inhibition of proliferation, migration and capillary-like formation of ox-LDL-exposed HAECs. Besides, our study showed that circ_0003204 in plasma EVs served as a potential biomarker for diagnosis and prognosis of cerebral atherosclerosis.

## Materials and methods

### Study population

From April to December 2018, a total of 67 individuals were recruited from the First Affiliated Hospital of Shandong First Medical University, and categorized into cerebral atherosclerosis group (*n* = 35; 18 males and 17 females; mean age = 65.18 ± 11.93) and control group (*n* = 32; 17 males and 15 females, mean age = 60.76 ± 10.91). The inclusion criteria of patients was described as previous study with a little modification [18]. Briefly, all the patients were examined by MRI or CT to exclude any previous history of stroke. Atherosclerosis and angiostenosis were assessed through examination of cerebrovascular TCD/MRA/CTA. Patients with cerebral atherosclerosis and vascular stenosis greater than or equal to 50% were included in the cerebral atherosclerosis group. The subjects without atherosclerosis or vascular stenosis less than 50%, were selected as control group. We excluded all subjects that could be diagnosed as these disorders following below, such as severe heart disease, stroke, intracranial hemorrhage, dissection, vasculitis, severe infections, nephrosis disease, liver disease, thrombotic diseases and tumors. Baseline characteristics were documented at the time of admission, including age, gender, history of diabetes mellitus (DM), smoking, drinking and hypertension. Laboratory parameters were also derived, including triglyceride (TG), total cholesterol (TC), low-density lipoproteincholesterol (LDL-C), high-density lipoprotein cholesterol (HDL-C), homocysteine level and Lipoprotein phospholipase A2. Hypertension was defined as resting systolic blood pressure ≥ 140 mmHg and/or diastolic blood pressure ≥ 90 mmHg. Diabetes was defined as fasting blood glucose ≥7.0 mmol/L or a diagnosis of diabetes needing diet. Individuals who formerly or currently smoked more than 6 months or daily smoked more than 20 cigarettes were defined as smokers. Excessive drinking is defined as drinking alcohol more than 25 g/day for adult males and more than 15 g/day for adult females. These subjects were followed until time to event or, in the case of no event, until August 2019. The end event was a composite outcome of stroke, transient ischemic attack (TIA), major vascular events and mortality. The diagnosis of stroke and TIA was defined according to the American Heart Association/American Stroke Association guideline [19]. The mortality was defined as cerebrovascular death. The follow-up rate was 91%. This study was reviewed and approved by Institutional Review Board of the First Affiliated Hospital of Shandong First Medical University, and patient consent was acquired prior to the initiation of experiment.

### Cell culture

HAECs was purchased from ScienCell (Carlsbad, CA, USA). The cells were cultured in endothelial cell medium supplemented with 10%FBS, 1% endothelial cell growth supplement (ECGS), 100 IU/ml penicillin, 0.1 mg/ml streptomycin (ScienCell) at 37 °C in a humidified atmosphere of 5% CO2. Confluent HAECs were maintained for 48 h with or without the presence of ox-LDL (50μg/mL; Beijing Solarbio Life Science Company) for further study.

### EVs isolation

EVs were extracted from HAEC cell culture medium or plasma samples using an ExoQuick precipitation kit (SBI, System Biosciences, Mountain view, CA) according to the manufacturer’s instructions. Briefly, the culture medium and plasma were thawed on ice and centrifuged at 3000×g for 15 min and 10,000×g for 30 min. For plasma EV isolation, 250 μl of the supernatant was mixed with 67 μl of the ExoQuick precipitation reagent and incubated at 4°Cfor 30 min, followed by centrifugation at 3000×g for 10 min. For the isolation of EVs in cell medium, an Amicon Ultra Centrifugal Filter Unit (100 kDa, Millipore) was used to concentrate the supernatant. The ultrafiltration supernatant was mixed with the ExoQuick precipitation reagent at the ratio of 5:1, and incubated at 4 °C overnight, followed by centrifugation at 1500×g for 30 min. The EV pellet was subsequently resuspended in 200 μl phosphate buffered saline (PBS). This isolation method has been well validated with other techniques including electron microscopy [20]. EV concentrations and size distribution were measured by nanoparticle tracking analysis (NTA) (NanoSight, NanoSight Ltd., UK).

### CCK-8 proliferation vitality assay

Cell viability was measured using the Cell Counting Kit 8 (Dojindo, Shanghai, China) according to the manufacturer’s instructions. HAECs were seeded into a 96-well plates at a density of 5 × 10^3^ cells/well at 37 °C. The cell viability was measured at the time point using microplate reader (Bio-Rad) by spectrophotometry at 450 nm.

### Migration assay

The migration of HAECs was determined using a 24-well modified Boyden chamber(8 μm, Corning). Approximately 5 × 10^4^ cells in 0.3 ml serum-free medium were added in the upper chamber. 0.6 ml medium with 10% FBS was seeded in the lower chamber as a chemoattractant. Following 24 h of incubation, the cells on the lower side of the chamber were fixed in 4% paraformaldehyde for 20 min and dyed with 0.1% crystal violet staining solution (Beyotime, Nantong, China) for 10 min, and then were counted and photographed in five representative fields. All experiments were repeated three times independently.

### Wound healing assay

Cell motility was assessed by performing a wound-healing assay. Cells were cultured in 6-well plates (5 × 10^4^ cells per well). At 80–90% confluence, the monolayer of cells was scratched using a sterile 200 μL tip, and then, cells were cultured under standard conditions for 24 h. Following several washes, recovery of the wound was captured at 0 and 24 h in a phase contrast microscope. All experiments were carried out in triplicate.

### Tube formation assay

Capillary-like network formation was performed to detect the angiogenic ability of HAECs. Briefly, HAECs were seeded at a density of 2 × 10^4^ on 96-well plates coated with 60 μL Matrigel (BD Bioscience). Being cultured for 48 h, the average number of capillary-like branches was counted in 5 random microscopic fields with a computer-assisted microscope.

### Plasmid, siRNAs and miRNA mimic and inhibitor

Plasmid of circ_0003204 overexpression, siRNA targeting circ_0003204 and non-specific negative control were purchased from RiboBio (Guangzhou, China). The microRNA mimics/inhibitor and corresponding negative control for miR-370-3p as well as TGFβR2 siRNA were also purchased from RiboBio. The sequences of circ_0003204 siRNA, TGFβR2 siRNA and its negative control were shown in Additional file 1: Table S1. HAECs were planted in 6-well plates 24 h prior to circ_0003204 vector, miR-370 mimic or inhibitor transfection with 50–60% confluence, and then were transfected using Lipofectamine™ RNAiMax (Invitrogen) according to the manufacture instructions.

### Sanger sequencing

The amplification products were inserted into a T-vector for Sanger sequencing to determine their full-length. The primers were synthesized in RiboBio, and Sanger sequencing was performed by Biorui (Beijing, China).

### Quantitative real-time PCR (qRT-PCR)

Total RNA was extracted extracted from EVs or cell samples using TRIzol (Thermol Fisher Scientific, MA, USA) and reverse transcription was performed using miScript II RT Kit (Qiagen, MD, USA) and cDNA amplification using the SYBR Green Master Mix kit (Takara, Otsu, Japan). The reverse transcription of circRNAs were performed using a HiScript Q RT SuperMix for qPCR Kit (Vazyme, Naijing, China) and quantified using SYBR Green Real-time PCR Master Mix. The nuclear and cytoplasmic fractions were isolated using NE-PER Nuclear and Cytoplasmic Extraction Reagents (Thermol Fisher Scientific, MA, USA). All of the primers were synthesized by RiboBio and listed in Additional file 1: Table S1.

### Western blot

Proteins were extracted from EVs and cells using RIPA Lysis and Extraction Buffer (Thermo Fisher Scientific, MA, USA) containing Protease/Phosphatase Inhibitor Cocktail (Abcam, Cambridge, MA, USA). The extracted proteins were separated in 10% SDS-polyacrylamide gel, and then transferred to immobilon-P membranes (Merck Millipore, Darmstadt, Germany). The membranes were blocked with 5% w/v Bovine Serum Albumin (Sigma-Aldrich, MO, USA), followed by incubation overnight with primary antibodies as follows: anti-FLOT-1 (1:1000, Cell Signaling Tech, MA, USA), anti-CD63 (1:2000, Abcam), anti-TGS101 (1:1000, Abcam), anti-TGFβR2 (1:1000, Abcam), anti-SMAD3 (1:1000, Cell Signaling Tech) and anti-phosph-SMAD3 (1:1000, Cell Signaling Tech). The membranes were then incubated with secondary antibodies (1:2000, HRP-linked anti-Rabbit IgG, Cell Signaling Tech), and digital images were visualized with the use of an Immobilon Western Chemiluminescent HRP substrate (Millipore, Darmstadt, Germany).

### Actinomycin D and RNase R treatment

Transcription was inhibited by the addition of 2 mg/ml Actinomycin D or DMSO (Sigma-Aldrich, St. Louis) as the negative control. Total RNA (5 μg) was incubated for 30 min at 37 °C with 4 U/μg of RNaseR (Epicentre Biotechnologies). After treatment with Actinomycin D and RNase R, the expression levels of USP36 mRNA and circ_0003204 were detected by qRT-PCR.

### FISH analysis

HAECs cultured on coverslips were fixed with 4% PFA for 10 min and incubated in PBS overnight at 4 °C, followed by processing to detect circ_0003204 or miR-370 expression. Next, the cells were permeabilized with 0.5% Triton X-100 in PBS for 15 min. After dehydration with 70, 95 and 100% ethanol for 5 min, hybridization buffer containing a Cy3-labeled circ_0003204 probe (RiboBio, Guangzhou, China) and a FITC-labeled miR-370 probe (RiboBio, Guangzhou, China) was heated to 88 °C for 5 min and dripped onto the coverslips, followed by hybridization at 37 °C overnight in a dark moist chamber. The next day, the coverslips were washed three times in 2X SSC (the first time at 42 °C, the rest at room tempture). The signals of the probes were detected by Fluorescent In Situ Hybridization Kit (RiboBio, Guangzhou, China) according to the manufacturer’s instructions. Then, the coverslips were washed three times with PBS and incubated with DAPI (Santa Cruz Biotechnology) for 20 min at room temperature to visualize nuclei. The sections were finally mounted with rubber cement. Immunofluorescence images were captured via microscopy (Leica, Germany). The circ_0003204 and miR-370 probe sequences were seen in Additional file 1: Table S1.

### RIP assay

RIP was performed using a Magna RIP Kit (Millipore, Billerica, MA, USA) following the manufacturer’s instructions. The abundance of miR-370 and circ_0003204 was tested using qRT-PCR. The antibodies against Ago2 and IgG used for RIP were purchased from Abcam.

### Luciferase activity assay

HEK-293 T cells were seeded in 96-well plates and cultured to 50–70% confluence before transfection. The constructs containing wild-type or mutant circ_0003204-miR-370 were inserted into luciferase gene by psiCHECK-2 vector as well as TGFβR2-miR-370 by a pmirGLO vector (Promega Corporation, Madison, WI, USA). 100 ng of luciferase reporter vectors and 20 pmol of miR-370 mimics/NC were transfected to 293 T cells for 24 h by Lipofectamine 2000. After 24 h incubation, the Promega Dual-Luciferase system was used to detect firefly and Renilla luciferase activities. The ratios of firefly to Renilla luciferase activities were calculated and repeated three times to determine relative luciferase activity.

### Microarray data

The gene expression profiles of GSE13139, GSE28829, GSE34645, GSE34644 and GSE34646 were downloaded from Gene Expression Omnibus (GEO, http://www.ncbi.nlm.nih.gov/geo). GSE13139 and GSE28829 were performed on GPL570: [HG-U133_Plus_2] Affymetrix Human Genome U133 Plus 2.0 Array while GSE34645, GSE34644 and GSE34646 on GPL15053: Applied Biosystems Taqman Array Rodent MicroRNA Cards v2.0. We extracted part of data from GSE13139 for further analysis, including 3 sample of ox-LDL treatment and 3 control samples.

### Data preprocessing and differently expressed gene (DEG) screening

The downloaded platform and series of matrix files were converted using the R language software and annotation package. The ID corresponding to the probe name was converted into an international standard name for genes (gene symbol). Gene differential expression was performed using the limma package in R, with treated samples verse untreated ones. Multiple testing correction was done to control the overall error rate using the Benjamini-Hochberg false discovery rate (FDR). An FDR < 0.05 and a |log_2_ Fold Change (FC)| > 2 were used as the cut-off criterion to identify the final DEGs.

### Bioinformatics analysis

We identified the predicted miRNAs targeting circ_0003204 using a bioinformatic programs: Circinteractome (http://circinteractome.nia.nih.gov). The overlapped target microRNAs of significantly upregulated genes from GSE13139 and GSE28829 were predicted using combination of Targetscan (http://targetscan.org), miRDB (http://mirdb.org) and miRanda (http://microrna.org). GSEA (http://software.broadinstitute.org/gesa/) was performed to investigate Kyoto Encyclopedia of Genes and Genomes (KEGG) pathways of upregulated gene expression in GSE13139. Selected enriched pathways had a relaxed FDR < 0.25 and *P* < 0.005. Gene Ontology (GO) and KEGG pathways analysis were performed to predict the potential functions of genes associated with circ_0003204 and upregulated genes with log_2_FC > 2 and *P*-value < 0.05 in GSE13139 using the Metascape bioinformatics tool (http://metascape.org). Only terms with P-value < 0.05, minimum count of 3, and enrichment factor of > 1.5 were considered as significant. A subset of enriched terms was selected and rendered as a network plot to further determine the relationship among terms, where terms with similarity of > 0.3 were connected by edges. Protein–protein interaction enrichment analysis was performed using the following databases: BioGrid, InWeb_IM, and OmniPath. Further, Molecular Complex Detection (MCODE) algorithm was applied to identify densely connected network components. Topology analysis was used to analyze the connectivity of the nodes in the PPI network to obtain a higher degree of key nodes. The hub genes were selected as ‘degree > 6’ for further analysis. Functional enrichment analysis of each module was performed using Metascape, with a significance threshold of *P* < 0.01.

### Statistical analysis

Statistical analyses were carried out by using SPSS 17.0 (IBM, SPSS, Chicago, IL, USA) and GraphPad Prism 7.0. All continuous variables were expressed as mean ± standard deviation (SD) or median (interquartile range). The chi-square test or Fisher’s exact test was used to express categorical variables. Two treatment groups were compared by the unpaired Students t test. Non-normallydistributed data were compared using Mann-Whitney U test andKruskal-Wallis test. Statistical difference between three or more were determined by a one-way analysis of variance. Multivariable logistic regression analysis was performed while evaluating the relationship between cerebrovascular atherosclerosis and related risk factors. The predictive function for distinguishing cerebral atherosclerosis and control group was characterized by ROC, and area under ROC curve (AUC) was calculated for assessing the diagnostic performance of selected markers. The Spearson’s correlation coefficient analysis was used to analyze the correlations. Event-free curves were analyzed with the Kaplane-Meier method and log-rank test. *P* < 0.05 was considered statistically significant.

## Results

### Identification and characteristics of circ_0003204 in HAECs

Mounting evidence shows that circRNAs as a novel type of ncRNAs could sponge miRNAs, regulate gene transcription and interact with RBPs involved in atherosclerosis [21]. Microarray analysis of circRNA in previous study revealed that circ_0004543 and circ_0003204 expression in HUVECs are significantly increased with treatment of ox-LDL [17], but it remained unclear for these two circRNAs level in ox-LDL-treated HAECs. QRT-PCR analysis indicated that treatment of HAECs by 50 μg/ml ox-LDL for 24 h could promote circ_0003204 expression in HAECs rather than circ_0004543 (Fig. 1a). Subsequently, we noted that circ_0003204 (chr17:76,798,405–76,800,060) is derived from exon 16 and 17 regions within ubiquitin specific peptidase 36 (USP36) locus (Fig. 1b). The genomic position revealed that the 16th and 17th exons from the USP36 gene are intermediated by long introns (Fig. 1b). Compared with the linear USP36 based on the qRT-PCR analysis, circ_0003204 had a resistant ability against digestion induced by RNase R exonuclease, indicating that circ_0003204 harbors a loop structure (Fig. 1c). We next observed the stability and localization of circ_0003204. After treatment with Actinomycin D, an inhibitor of transcription at the indicated time points, total RNA was separated from HAECs. QRT-PCR analysis showed that the transcript half-life of circ_0003204 exceeded 24 h, while that of linear USP36 displayed about 6 h in HAECs (Fig. 1d), indicating that circ_0003204 is highly stable in HAECs. Cytoplasmic and nuclear RNA analysis of qRT-PCR uncovered that circ_0003204 was preferentially localized in the cytoplasm in HAECs (Fig. 1e). Furthermore, FISH was used to assess circ_0003204 localization in HAECs showing that circ_0003204 (red fluorescent distribution) was mainly localized in the cytoplasm of HAECs (Fig. 1f). Collectively, these results suggested that circ_0003204 is a highly stable and cytoplasmic circRNA derived from the USP36 gene locus.

**Fig. 1:** Validation and characteristics of circ_0003204 in HAECs. **a** The expression of circ_0003204 and circ_0004543 in HAECs treated by ox-LDL (50μg/ml) for 24 h. **b** Schematic illustration showing USP36 exons 16–17 circularization to form circ_0003204 (black arrow). The presence of circ_0003204 was validated by qRT-PCR, followed by Sanger sequencing. The red arrow represents head-to-tail circ_0003204 splicing sites. **c** QRT-PCR analysis for circ_0003204 expression in HAECs treated with or without RNase R digestion. The relative expression of circ_0003204 and USP36 mRNA were normalised to the values measured for mock treatment. **d** QRT-PCR analysis of circ_0003204 and USP36 mRNA in HAECs treated with Actinomycin D at the indicated time points. **e** QRT-PCR analysis of circ_0003204 and USP36 mRNA in the cytoplasm or the nucleus in HAECs. **f** FISH indicated the localization of circ_0003204 in the cytoplasm. Cytoplasmic circ_0003204 probe was stained with Cy3 for red color. Nuclei were stained with DAPI for blue color. Scale bar = 20 μM. DAPI, 4′,6-diamidino-2-phenylindole; FISH, fluorescence in situ hybridization; qRT-PCR, real-time quantitative PCR. The values are expressed as mean ± SD from three independent experiments, *P < 0.05

### Circ_0003204 inhibits the HAECs proliferation, migration and tube formation in vitro

To identify the biological functions of circ_0003204 in the regulation of HAECs phenotype, we transfected HAECs with circ_0003204 overexpresson (OE) vector and small-interfering RNA (siRNA), and then examined the expression level of circ_0003204 (Fig. 2a). Then we found that knockdown of circ_0003204 had little effect on USP36 mRNA level in HAECs (Fig. 2b). Subsequently, cell viability assay was carried out to reveal that overexpression of circ_0003204 inhibited growth of HAECs, while knockdown of circ_0003204 reversed the repressive effects of circ_0003204 overexpression (Fig. 2c and d). Then, transwell and scratch assays demonstrated that circ_0003204 OE could aggravate low mobility of ox-LDL- treated HAECs while circ_0003204 knockdown alleviated impaired motility of HAECs ox-LDL caused (Fig. 2e and f), which was analogous to the impact of circ_0003204 on control HAECs (Fig. 2e). In addition, we dissected capillary network formation of ox-LDL-treated HAECs as well as control treatment, which uncovered that circ_0003204 acted like antagonist against tube formation of HAECs (Fig. 2g). Taken together, our results implied the involvement of circ_0003204 in the regulation of HAECs ectopic phenotype ox-LDL caused.

**Fig. 2:** The effects of circ_0003204 on HAEC proliferation, motility and tube formation. **a** QRT-PCR analysis of the transfection efficiency of circ_0003204 overexpression or si-circ_0003204 after transfection for 48 h in HAECs. **b** QRT-PCR analysis of USP36 mRNA level normalised to GAPDH after transfection with circ_0003204 siRNA or negative control into HAECs for 48 h. **c** and **d** Cellular viability analysis of HAECs transfected with circ_0003204 overexpression vector or circ_0003204 siRNA using CCK-8 assay. **e** Analysis of cell migration potential of HAECs transfected with circ_0003204 overexpression or si-circ_0003204 vectors using transwell assay. Scale bar = 25 μm. **f** Wound healing assay for analysis of ox-LDL-exposed HAECs migration after transfection of circ_0003204 overexpression or si-circ_0003204 vectors. Scale bar = 50 μm. **g** Analysis of vasculogenesis ability of HAECs transfected with circ_0003204 overexpression or si-circ_0003204 vectors. Scale bar = 100 μm. OE, overexpression; siRNA, small interfering RNA; NC, negative control; CTL, control. Data are the means ± SD of three experiments. *P and **P < 0.05

### Circ_0003204 acts as a miRNA sponge for miR-370

Given that circ_0003204 played a critical role in the regulation of HAEC phenotype, we thus uncovered the underlying mechanisms for circ_0003204. We first downloaded microarray data from GEO datasets (GSE13139) and performed bioinformatic analysis of gene profiles referred to ox-LDL-treated HAECs. The heating cluster map revealed significant changes of DEGs in ox-LDL-treated HAECs compared with their expression in the sham group (Fig. 3a). Figure 3b was indicative of normalization of GSE13139. The variation of gene expression between the sham and ox-LDL treated was shown in volcano and scatter plots in Fig. 3c and d. Of these genes, 88 with log_2_FC >2 and *P* < 0.05 were considered to be significantly upregulated, and 98 with log_2_FC < -2 and P < 0.05 were significantly downregulated. We then performed GO and pathway analysis of these 88 upregulated genes to speculate the potential functions of upregulated circRNAs as indicated in Additional file 1: Figure S1, for instance, one of the enriched KEGG for the upregulated genes, cAMP signaling pathway, has been confirmed to be involved in the progression of atherosclerosis [22]. In the one hand, it is well-established that circRNAs could act as an endogenous RNA sponge to interact with miRNAs and influence the expression of targeted genes [23]. We therefore investigated which miRNAs circ_0003204 sponges. Bioinformatics programme circinteractome predicted 39 miRNAs which could bind to the recognition seed in circ_0003204 sequence, and circ_0003204/39 downstream miRNAs/mRNA interaction network was shown in Additional file 1: Figure S2. Subsequently, the combination of Targetscan, miRanda and miRDB predicted 106 candidate miRNAs which could bind to 3′ UTR of 88 significantly upregulated genes in GSE13139 (Fig. 3e). Six miRNAs were selected through overlapping these two datasets (Fig. 3e). To further investigate whether circ_0003204 was involved in the progression of atherosclerotic plaques, the upregulated DEGs in GSE28829 were used to predict 133 targeted miRNAs using Targetscan, miRanda and miRDB, and then 39 circinteractome-predicted miRNAs for circ_0003204 were overlapped with these 133 targeted miRNAs, which displayed 7 overlapped miRNAs (Fig. 3f). Subsequently, to speculate the potential functions of circ_0003204, we performed GO and pathway analysis of these 13 overlapped miRNAs (6 in Fig. 3e and 7 in Fig. 3f) and their PPI network involved in atherosclerosis (Additional file 1: Figure S3). The enriched KEGG pathways, including AMPK signaling pathway and FOXO signaling pathway (Additional file 1: Figure S3D), have been confirmed to be involved in the progression of atherosclerosis [24, 25]. In addition, notably, both hsa-miR-370 and hsa-miR-197 were enriched into the overlapped miRNAs in Fig. 3e and f. Due to the miRNA conserved property between mouse and human, the expression level of both mmu-miR-370 and mmu-miR-197 were further detected in miRNA profiles GSE34645, GSE34644 and GSE34646. As indicated in Additional file 1: Figure S4A and B, the expressions of mmu-miR-370 in early atherosclerosis plaque significantly fell down to less than 50% of non-atherosclerosis artery tissue (*P* < 0.05), but no statistical significance was found in mmu-miR-197 expression between them, despite the downregulated expression of mmu-miR-197 in the early atherosclerosis plaque. Intriguingly, the expression of mmu-miR-370 and mmu-miR-197 in advanced atherosclerosis plaque remained unchanged (Additional file 1: Figure S4C and D). More importantly, miR-370 was the only candidate microRNA after overlapping circinteractome-predicted miRNAs for circ_0003204 with the significantly downregulated microRNAs in GSE34645 (Fig. 3g). These results suggested that miR-370 was involved in the early development of atherosclerotic plaque. Moreover, literature reviews of miR-370 have shown that miR-370 could be downregulated by ox-LDL dose-dependently and time-dependently, which induces the increase of IL-6 and IL-1β [26], whereas miR-370 overexpression had positive impact on the invasion and proliferation of HUVECs [27]. Therefore, we constructed a circ_0003204 fragment and incorporated it into downstream of the luciferase reporter gene and hypothesized that miR-370 could reduce the luciferase activity of circ_0003204 (Fig. 3h). Luciferase assay confirmed that site 1 of miR-370 was able to result in the lower luciferase reporter activity compared with site 2, indicating that miR-370 might have potential to bind with circ_0003204 (Fig. 3i), then we found that circ_0003204 and miR-370 were more abundant in Ago2 pellet than in the IgG pellet (Fig. 3j). Subsequently, we performed FISH assay to reveal that circ_0003204 and miR-370 colocalized in the cytoplasm (Fig. 3k). Additionally, it was demonstrated that miR-370 expression in HAECs could be inhibited by ox-LDL (Fig. 3l). Given that circ_0003204 was able to bind with miR-370, we then detected the expression level of miR-370 via gain/loss-of-function of circ_0003204, indicating decreased expression of miR-370 concomitant with circ_0003204 overexpression while increased expression of miR-370 with circ_0003204 inhibition (Fig. 3m), but miR-370 mimics or inhibitor had no impact on the expression of circ_0003204 (Fig. 3n).

**Fig. 3:** Circ_0003204 serves as a sponge for miR-370 in HAECs. **a** A microarray heat map from GSE13139 representing discrepant mRNA expression values in HAECs treated by ox-LDL (50μg/ml) for 24 h compared with those treated by control (fold change > 2, P< 0.05). **b** The standardization of differently expressed mRNAs in GSE13139. **c** A volcano plot presenting the differently expressed mRNAs (|log_2_FC| > 2, *P* < 0.05) from GSE13139. **d** A scatter plot assessing mRNA expression variation between the sham and ox-LDL-treated group from GSE13139. **e** Schematic illustration showing the overlap between the predicted miRNAs for circ_0003204 by Circinteractome and the predicted miRNAs for upregulated DEG using the combination of Targetscan, miRanda and miRDB. **f** Schematic illustration showing the overlap between the predicted miRNAs for circ_0003204 using Circinteractome and the predicted miRNAs for significantly upregulated DEGs from GSE28829 using Targetscan, miRanda and miRDB. **g** Schematic illustration showing the overlap between the predicted miRNAs for circ_0003204 using Circinteractome and the significantly downregulated miRNAs in GSE34645. **h** Schematic representation of two complementary binding sites of circ_0003204 with miR-370. **i** Luciferase activity of cotransfection of circ_0003204 and miR-370 mimics/negative control. **g** RIP indicated the correlation of circ_0003204 and miR-370 with Ago2. Ago2 protein was tested by IP-western blot, and the expression of circ_0003204 and miR-370 were investigated using qRT-PCR. **k** FISH assay showed the location of circ_0003204 and miR-370 in HAECs. Red, circ_0003204; Green, miR-370; Blue, DAPI. Scale bar = 20um. **l** QRT-PCR analysis showing the effect of ox-LDL on miR-370 level in HAECs. **m** MiR-370 expression in ox-LDL-treated HAECs measured by qRT-PCR after circ_0003204 overexpression or knockdown. **n** Circ_0003204 expression in ox-LDL-treated HAECs measured by qRT-PCR after miR-370 overexpression or knockdown. NC, negative controk; WT, wild type; MT, mutant; DAPI, 4′,6-diamidino-2-phenylindole; FISH, fluorescence in situ hybridisation; CTL, control; OE, overexpression; siRNA, small interfering RNA. Data are means ± SD of three experiments. *P and **P < 0.05.

### TGFβR2 is a target gene of miR-370

Previous studies have confirmed that FOXO1 was identified as functional target of miR-370, which could prohibit the invasion and proliferation of human umbilical vein endothelial cells [25]. However, little is known about which signaling pathway miR-370/FOXO1 was involved in. KEGG analysis showed that FOXO1 was enriched into pathways in cancer, AMPK signaling pathway, FOXO signaling pathway, prostate cancer and insulin resistance, etc., all of which remarkably overlapped signaling pathways of circ_0003204 (Additional file 1: Figure S3D). in addition, it was found that FOXO pathway was involved in endothelial protection against atherosclerosis [28], in which TGFβR2, a predictive target of miR-370 by combination of Targetscan, miRDB and miRanda, was involved as well [29] (Additional file 1: Figure S5). Interestingly, TGFβR2 was found to participate in TGFβ signaling pathway [30] with which signaling pathways of circ_0003204 also shared (Additional file 1: Figure S2D). Accordingly, it may speculate that the alternation in miR-370/TGFβR2 axis might underlie the biological function of circ_0003204. To investigate this hypothesis, TGFβR2 was selected to demonstrate whether it can directly bind with miR-370. Firstly, miR-370 mimic or inhibitor were respectively transfected into ox-LDL-treated HAECs. After transfection for 48 h, qRT-PCR and western blot analysis displayed low expression of TGFβR2 in HAECs after miR-370 mimics transfection (Fig. 4a and b), and conversely, high expression of TGFβR2 with miR-370 inhibitor (Fig. 4c and d). Figure 4e represented the potential binding sites of wild type or mutant TGFβR2 with miR-370. Additionally, the luciferase activity of wild type TGFβR2 3’UTR was evidently decreased in miR-370 mimic group, However, the luciferase activity of mutant TGFβR2 3’UTR remained unchanged after transfection of miR-370 mimic (Fig. 4f).

**Fig. 4:** TGFβR2 is the downstream target of miR-370. **a** and **c** QRT-PCR analysis of TGFβR2 expression after transfection of miR-370 mimics or inhibitor to ox-LDL-treated HAECs for 48 h. **b** and **d** Western blot analysis of TGFβR2 protein expression after transfection of miR-370 mimics or inhibitor to ox-LDL-treated HAECs for 48 h. **e** Putative miR-370 binding sites in TGFβR2. The predictive complementary sequences are indicated in red. **f** Relative luciferase activity of wild-type and 3’UTR mutant constructs of TGFβR2 cotransfected with miR-370 mimics and miRNA negative control. NC, negative control; UTR, untranslated regions. Data are means ± SD of three experiments. *P < 0.05

### Circ_0003204/miR0–370 axis blocks HAEC viability, migration and tube formation via downstream TGFβR2/phosph-SMAD3

To further exploit the functionality of miR-370/TGFβR2 axis in ox-LDL-treated HAECs, we performed function experiments, such as cell viability, motility and tube formation. It was demonstrated that the inhibitory effects of miR-370 knockdown on cell proliferation (Fig. 5a), cell motility (Fig. 5b and c) and capillary-like formation (Fig. 5d) were reversed by cotransfection of TGFβR2 siRNA. Subsequently, we detected phosph-SMAD3 protein expression in ox-LDL-treated HAECs after transfection of TGFβR2 siRNA. Western blot analysis displayed the decreased expression of phosph-SMAD3 after delivery of TGFβR2 siRNA into ox-LDL-treated HAECs (Fig. 5e). Then, SIS3, a specific phosph-SMAD3 inhibitor, was used to reveal that downregulation of phosph-SMAD3 protein evidently alleviated the impaired proliferation (Fig. 5f), migration (Fig. 5g and h) and capillary network (Fig. 5i) of HAECs with ox-LDL stimulation whereas inhibited these angiogenic responses of HAECs with control treatment. Next, we examined the protein expression of TGFβR2 and its downstream phosph-SMAD3 in ox-LDL-treated HAECs after cotransfection with circ_0003204 siRNA and miR-370 inhibitor (Fig. 5j), indicating that knockdown of circ_0003204 could inhibit the expression of TGFβR2 and phospho-SMAD3 protein via counteracting miR-370 inhibitor function. Moreover, knockdown of circ_0003204 could block the repressive effect of miR-370 inhibitor on cell viability (Fig. 5k), motility (Fig. 5l and m) and tube formation (Fig. 5n). Based on previous report that SMAD3 phosphorylation and nuclear translocation could be promoted by ox-LDL treatment, leading to deactivation of endothelial cell [31], our results suggested that circ_0003204 could exacerbate deactivation of HAECs in response to ox-LDL via miR-370/TGFβR2/phospho-SMAD3 axis.

**Fig. 5:** The circ_0003204/miR-370 axis could induce HAEC deactivation via its downstream gene TGFβR2. **a** Cell proliferation activity was measured by CCK-8 assay after transfection with TGFβR2 siRNA + miR-370 inhibitor into ox-LDL-treated HAECs. *P < 0.05 versus siRNA control cotransfected with inhibitor control group. **b** Cell motility was measured by transwell assay after transfection with TGFβR2 siRNA + miR-370 inhibitor into ox-LDL-treated HAECs. *P < 0.05. Scale bar = 25 μm. **c** Cell migration potential was detected by wound healing assay after transfection with TGFβR2 siRNA + miR-370 inhibitor into ox-LDL-treated HAECs. *P < 0.05. Scale bar =50 μm. **d** Tube formation was measured by Matrigel assay after transfection with TGFβR2 siRNA + miR-370 inhibitor into ox-LDL-treated HAECs. *P < 0.05. Scale bar = 100 μm. **e** Western blot analysis indicating phosph-SMAD3 and SMAD3 protein level after transfection with TGFβR2 siRNA into ox-LDL-treated HAECs. *P < 0.05. **f** Cell proliferation activity was measured by CCK-8 assay after SIS3 (3 μM) + ox-LDL (50 μg/ml) treatment. *P < 0.05. **g** Cell motility was measured by transwell assay after SIS3 (3 μM) + ox-LDL (50 μg/ml) treatment. *P < 0.05. Scale bar = 25 μm. **h** Cell migration was measured by wound healing assay after SIS3 (3 μM) + ox-LDL (50 μg/ml) treatment. *P < 0.05. Scale bar =50 μm. **i** Tube formation was measured by Matrigel assay after SIS3 (3 μM) + ox-LDL (50 μg/ml) treatment. *P < 0.05. Scale bar = 100 μm. **j** Western blot analysis showing TGFβR2 and phosph-SMAD3 expression after cotransfection of circ_0003204 siRNA + miR-370 inhibitor into ox-LDL-treated HAECs. *P and **P < 0.05. **k** Cell proliferation activity was measured by CCK-8 assay after transfection with circ_0003204 siRNA + miR-370 inhibitor into ox-LDL-treated HAECs. *P < 0.05 versus group with contransfection of circRNA-siRNA NC and miRNA-inhibitor NC. **l** Cell motility was measured by transwell assay after transfection with circ_0003204 siRNA + miR-370 inhibitor into ox-LDL-treated HAECs. *P < 0.05. Scale bar = 25 um. **m** Cell migration potential was detected by wound healing assay after transfection with circ_0003204 siRNA + miR-370 inhibitor into ox-LDL-treated HAECs. *P < 0.05. Scale bar =50 μm. **n** Tube formation was measured by Matrigel assay after transfection with circ_0003204 siRNA + miR-370 inhibitor into ox-LDL-treated HAECs. *P < 0.05. Scale bar = 100 um. NC, negative control; siRNA, small interfering RNA. Data are means±SD of three experiments

### Circ_003204 and miR-370 expression in the plasma EVs from the patients with cerebral atherosclerosis

Based on LiftOver tool in UCSC genome browser and CIRCpedia v2 database (http://www.picb.ac.cn/rnomics/circpedia/), there is no corresponding circRNA in the orthologous locus of mouse USP36 gene within 5-nt difference for hsa_circ_0003204. Consequently, the expression of mouse-derived circRNA analogous to hsa_circ_0003204 was undetectable in mouse tissue preventing studies in mouse models, such as middle cerebral artery occlusion. Therefore, we further explore circ_0003204 and miR-370 level in the clinical patients. In the present study, 35 patients with cerebral atherosclerosis and 32 control subjects were recruited into our study. Their demographic and clinical characteristics are provided in Additional file 1: Table S2. Since exosomes were demonstrated to play an essential role in cell-cell communication under various disease conditions, including atherosclerosis [29], we purified exosomes from the plasma of recruited subjects for detecting circ_0003204 and miR-370 expression. Most of the collected vesicles were typical in size as exosomes ranging from 50 nm to 150 nm (Fig. 6a), but some particles in diameter of < 50 nm or > 150 nm were also detected. Hence, these isolated vesicles were termed EVs rather than exosomes. Furthermore, these vesicles expressed characteristic exosome markers, such as FLOT-1 and CD63 (Fig. 6b). As anticipated from our results in vitro experiments, the expression of circ_0003204 in EVs from cerebral atherosclerosis patients was markedly higher compared with non-atherosclerosis groups (*P* < 0.05) (Fig. 6c). As for miR-370, it was found that the expression of miR-370 in EVs was lower in cerebral atherosclerosis patients compared with control group (0.91 ± 0.39 vs 1.14 ± 0.51), although no significant difference existed between them (*P* = 0.54) (Fig. 6d). To explore whether HAECs secreted EVs containing circ_0003204, we purified and isolated EVs from HAEC culture medium. The size distribution of EVs was detected using Nanosight, with a size peak of 103 nm (Fig. 6e). A western blot for exosome markers, such as CD63 and TSG101, further confirmed EVs identity (Fig. 6f). Importantly, it was found that the circ_0003204 level in EVs showed increasing tendency after HAECs were exposed to different concentration of ox-LDL (0–100 μg/ml) for 24 h (Fig. 6g). Then, HAECs were treated with ox-LDL stimulation (50μg/ml), and qRT-PCR assay showed an increased expression of circ_0003204 in EVs collected from culture medium at the indicated time points.

**Fig. 6:** Expression level of circ_0003204 and miR-370 in EVs for the cerebral atherosclerosis patients and healthy controls. **a** The size distribution of isolated EVs measured by nanoparticle tracking analysis. **b** Immunoblotting of EV markers using anti-CD63 and anti-FLOT-1 and β-actin as a loading control. **c** The circ_0003204 expression in EVs for cerebral atherosclerosis patients and healthy control as measured by qRT-PCR. *P < 0.05. **d** The expression level of miR-370 in EVs from cerebral atherosclerosis patients and healthy control. **e** Size distribution histogram of cell medium EVs by nanoparticle tracking analysis. **f** Immunoblotting of cell medium EV for CD63, TSG101 and β-actin. **g** QRT-PCR analysis of circ_0003204 expression in the cell medium EVs at the different concentration of ox-LDL (0–100 μg/ml). *P < 0.05. **h** QRT-PCR analysis of circ_0003204 expression in the EVs collected from HAECs with ox-LDL treatment (50 μg/ml) at the indicated time points. *P < 0.05. Data are means ± SD of three experiments

### The correlation of circ_0003204 expression in plasma EV and LDL-C level with cerebral atherosclerosis

As indicated in Additional file 1: Table S3, we found that circ_0003204 expression in the plasma EVs was positively related with cerebral atherosclerosis (r = 0.469, *P* < 0.001) (Fig. 7a) and LDL-C level (r = 0.299, *P* = 0.014) (Fig. 7b). Multivariate regression analysis revealed that both circ_0003204 in the plasma EVs and LDL-C level were correlated with cerebral atherosclerosis after adjusted for gender, age, history of drinking and smoking, TC, HDL-C, TG, hypertension, diabetes, HCY, Lp-PLA2 and miR-370 expression (Additional file 1: Table S4). In addition, ROC analysis was performed to predict the impact of circ_0003204 in the plasma EVs and LDL-C level on cerebral atherosclerosis. The AUC of circ_0003204 in the plasma EVs was 0.770 (95% CI 0.651–0.890; *P <* 0.001) (Fig. 7c), and the AUC of LDL-C level was 0.851 (95% CI 0.761–0.952; *P <* 0.001) (Fig. 7d). Notably, the AUC of the combination of circ_0003204 in the plasma EVs and LDL-C level was 0.875 (95% CI 0.777–0.954; *P <* 0.001*)* (Fig. 7e), suggesting that the combination of both had superior efficiency for predicting cerebral atherosclerosis than either circ_0003204 or LDL-C alone. To evaluate the association of circ_0003204 level in plasma EVs with the prognosis of recruited subjects, the patients with cerebral atherosclerosis and their healthy control were respectively divided into two groups on the basis of median value of circ_0003204 level: circ_0003204 high expression and circ_0003204 low expression. Kaplan Meier analysis illustrated that cerebral atherosclerosis patients with circ_0003204 high expression developed more frequent occurrence of end events compared with those with circ_0003204 low expression (log-rank *P* = 0.031) (Fig. 7f), but for these healthy control, the occurrence of end events had no significant difference between the subjects with circ_0003204 high expression and ones with circ_0003204 low expression (log-rank *P* = 0.197) (Fig. 7g). This may suggest that circ_0003204 in plasma EVs represented a prognostic factor for these events appearing in cerebral atherosclerosis patients.

**Fig. 7:** Correlation of circ_003204 in EVs and LDL-C level with cerebral atherosclerosis. **a** Spearson correlation coefficients between circ_0003204 and cerebral atherosclerosis. **b** Spearson correlation coefficients between circ_0003204 and LDL-C level. **c** ROC of circ_0003204 for cerebral atherosclerosis. **d** ROC of LDL-C for cerebral atherosclerosis. **e** ROC of combination of circ_003204 and LDL-C for cerebral atherosclerosis. **f** Kaplan-Meier analysis of the correlation of circ_0003204 expression level with occurrence of end events in cerebral atherosclerosis patients. **g** Kaplan-Meier analysis of the correlation of circ_0003204 expression level with occurrence of end events in non-atherosclerosis patients

## Discussion

Atherosclerosis triggered by multiple risky factor could cause severe cardio/cerebral-vascular disease, such as coronary heart disease, stroke and peripheral vascular disease. Aberrant differentiation and phenotypic transformation of EC are the critical initial steps contributing to atherosclerosis related vasculopathy [32]. Therefore, it is important to identify early biomarkers predicting endothelial differentiation and phenotype modification in atherosclerosis for prevention and treatment of such diseases. CircRNAs generated from exonic or intronic sequences are not only abundant in body fluids, but have more stable circular structure which is resistant to RNA exonuclease [13]. These characteristics provide circRNA better prospect for biomarker of human disease. Importantly, a growing amount of evidences have illustrated the association between circRNAs expression and atherosclerosis progress [21, 33], but little known is about the role of circRNA in endothelial phenotype involved in atherosclerosis. In this study, we verified increased expression of circ_0003204 in ox-LDL treated HAECs as well as EVs from HAEC culture media and plasma of the patients with cerebral atherosclerosis. Importantly, our study elucidated the involvement of circ_0003204-miR-370-TGFβR2 axis in atherosclerosis, especially, its role in endothelial phenotype alternation, suggesting that circ_0003204 might act as a therapeutic target for ox-LDL-induced ECs aberrant functions.

Differently expressed circRNAs have been reported to have important functions in buildup of atherosclerotic plaque [34]. For instances, as microRNA sponge, circCHFR, identified as a transcript at the locus of chromosome 12, serves as a stimulus for proliferation and migration of ox-LDL-induced VSMCs via sponging miR-370 [16]. Also, it was confirmed that circ_0044073 could favor proliferation and invasion of HUVECs and VSMCs by targeting miR-107 and activating its downstream JAK/STAT pathway against atherosclerosis [15]. Silencing of circWDR77 could alleviate proliferation and migration of high glucose induced VSMCs through miR-124/FGF2 axis [35]. As RBP, circANRIL was reported to induce apoptosis and alleviated proliferation of VSMC and macrophage via interaction with multiple RBPs for supervising pre-rRNA maturation and nucleolar stress [11]. In addition, Bazan HA et al. [36] discerned that the ratio of serum circR_284: miR-221 is significantly elevated in the early stage of carotid plaque rupture, implying its potential as diagnostic biomarker for carotid plaque rupture and stroke. In this current study, our results revealed elevated circ_0003204 expression in ox-LDL-treated HAECs as well as in EVs secreted from ox-LDL-treated HAECS and the plasma of cerebral atherosclerosis patients, which were partly line with previous study despite different EC types. Also, we demonstrated that circ_0003204 was not only characterized as an independent risky factor for atherosclerosis pathogenesis, but had potential diagnosis value for cerebral atherosclerosis. Additionally, it was found that cerebral atherosclerosis patients with higher expression of circ_0003204 were more likely to suffer end events. To our best knowledge, our study is the first to verify that circ_0003204 was a promising biomarker for assessing the diagnosis and prognosis of cerebrovascular atherosclerosis and stenosis. Larger cohort studies are required to further validate the relationship between circ_0003204 level and severity of cerebral vascular stenosis.

MiR-370, which was found to interact with circ_0003204 in our study, has been demonstrated to be an important microRNA in lipid metabolism which inhibits the expression of the carnitine palmitoyl transferase 1α gene regulating fatty acid oxidation [37]. Recent evidences have confirmed higher expression level of miR-370 in the plasma of hyperlipidemia patients with CAD as well as in the peripheral blood mononuclear cell of patients with coronary atherosclerosis [38]. Additionally, miR-370 was reported to modulate production of inflammatory factors (IL-6, IL-1β, et al.) and oxidative stress via targeting TLR4 in ox-LDL-incubated THP-1 cells [25]. However, few studies have assessed the role of miR-370 in the endothelial injury in atherosclerosis plaque. Similar with previous findings [16], bioinformatic analysis in the present study uncovered that miR-370 was predicted to be involved in the development and progression of atherosclerosis plaque. Subsequently, our in vitro experiment data indicated that miR-370 expression was decreased in HAECs treated with ox-LDL and that upregulation of miR-370 expression significantly promoted cellular proliferation, migration and capillary formation. Interestingly, we also found that miR-370 level was lower in the plasma EVs from cerebral atherosclerosis patients versus control subject in spite of no significant change observed, which was inconsistent with our in vitro results and previous studies [38]. The inconsistent findings about the association between miR-370 expression and atherosclerosis may be explained as follow: (1) discrepant clinical characters and experimental samples of patients among different studies. Our recruited population was a cohort of patients with cerebral vascular stenosis ≥50% due to atherosclerosis, irrespective of coronary artery atherosclerosis while other studies focused on CAD patients. In addition, in our study, miR-370 level was examined in purified EVs rather than in the whole plasma or serum. (2) different sample size among studies. Therefore, further studies are required to detect miR-370 level in EVs purified from larger cohort and elucidate the role of miR-370 in EVs.

Subsequently, to confirm whether miR-370 acted as a regulator for circ_0003204-related EC phenotype, circ_0003204 OE vector with miR-370 mimics were cotransfected into ox-LDL-treated ECs. We found that overexpression of miR-370 counteracted aberrant changes of EC phenotype circ_0003204 induced. These results suggested that miR-370, as a downstream target circ_0003204 sponged, was involved in endothelial phenotype mediated by circ_0003204. Also, our study indicated that miR-370 and its targeted gene TGFβR2 had notable impact on endothelial phenotype in atherosclerosis. TGFβR2, as one of three types of TGFβ receptors, can bind TGFβ ligand by autophosphorylation for cooperating with TGFβR1, which turns out phosphorylation and activation of downstream SMAD2 and SMAD3 [39]. Phosphorylated SMAD2/SMAD3 combine with SMAD4 protein forming hetero-oligomeric complexes, which translocated into nuclear to change transcription level of multiple genes, affecting biological characteristics of chronic inflammation, tumor and autoimmune reactions [40–42]. For instance, activated TGFβR2 could aggravate renal fibrosis by upregulating the expression of collagen 1 and α-smooth muscle actin [43]. In our study, we identified a new regulatory mechanism underlying TGFβR2 which acted as a downstream target of circ_0003204. Our research demonstrated that TGFβR2 played a pivotal role in EC proliferation, migration and capillary formation through the regulation of p-SMAD3, which positively supported our hypothesis that circ_003204/miR-370/TGFβR2 axis could regulate ectopic EC phenotype ox-LDL caused.

Several limitations should be noted in our study. Firstly, the detailed mechanism by which circ_0003204-miR-370-TGFβR2/phosph-SMAD3 axis mediates endothelial phenotype, especially which downstream targeted genes were directly or indirectly influenced by this axis, needs to be further validated in future studies. Secondly, due to no conserved property for circ_0003204 between species, the expression and function of circ_0003204 involved in the developmental and pathological angiogenesis were unable to be examined in mouse model. In addition, the main cell origin for circ_0003204 in plasma EVs was required to explore further, although our present results revealed that circ_0003204 was released into EVs in the conditioned medium of ox-LDL-treated HAECs. Our ongoing experiments will mainly focus on the comparison of circ_0003204 level among plasma neuron-derived EVs, glia cell-derived EVs, astrocyte-derived EVs, endothelial cell-derived exosomes and platelet-derived EVs. Lastly, the number of recruited subjects was limited, and thus circ_0003204, as a biomarker for diagnosis and prognosis of cerebrovascular atherosclerosis and stenosis should be further confirmed in other population groups, and the diagnostic and therapeutic value of EVs, especially miRNAs in EVs, for cerebrovascular atherosclerosis is required to be explored in large sample size.

## Conclusion

Summarily, our study disclosed regulatory mechanism of circ_0003204 that mediates endothelial phenotype through targeting miR-370-3p/TGFβR2/phosph-SMAD3 pathway (Fig. 8). Blockage of circ_0003204 is regarded as a potential therapeutic target for alleviation of EC aberrant phenotype in atherosclerosis pathology.

**Fig. 8:** Schematic illustration of the molecular mechanism of circ_0003204 underlying HAEC injury in atherosclerosis. Circ_0003204 regulated the miR-370/TGFβR2/phosph-SMAD3 axis by sponging miR-370 in HAECs. Increased expression of circ_0003204 in ox-LDL-treated HAECs inhibited miR-370 expression, which upregulated TGFβR2 and phosph-SMAD3 expression, thereby blocking the proliferation, migration and capillary formation of HAECs

## Supplementary information

**Additional file 1: Figure S1.** GO and pathway analysis of the upregulated genes in GSE13139. Dot plot representing biological process with the top 10 most significantly enriched terms (A), cellular component (B), molecular function (C), KEGG pathways (D) and Reactome pathways (E) for the upregulated genes. (F) GESA was conducted to search significant KEGG pathway for the upregulated genes. *P* < 0.001, FDR = 0.181. **Figure S2.** CircRNA-miRNA-mRNA network of hsa_circ_0003204 (red rhombic node) and its 39 predicted miRNAs (orange triangle nodes) and 10 highest-ranking candidate mRNAs (blue circular nodes). **Figure S3.** GO, KEGG and PPI network analysis of circ_0003204. Dot plot showing biological process (A), molecular function (B), cellular component (C) and KEGG (D) with the respective top 10 most significantly enriched terms. (E) Analysis of PPI network using Integrated Interactions Database with filter interaction by 'experimental and predicted' and 'atherosclerosis'. The hub genes in PPI was labeled with the colored nodes of which the color depth referred to the 'degree' calculated by Cytoscape. (F) KEGG enriched cluster of genes from PPI network using Metascape. (G) The genes in Fig.F were colored by their P-value. (H) The enriched cluster showing interaction of 7 modules in PPI network as analyzed by Metascape. (I) Seven modules obtained from PPI network. **Figure S4.** The expression level of mmu-miR-370 and mmu-miR-197 in GSE34645, GSE34644 and GSE34646. (A) A microarray heat map from GSE34645 representing discrepant miRNA expression in atherosclerosis plaque on 3 month high fat diet compared with undieased arterial tissue (|log2FC| > 2, *P* < 0.05). mmu-miR-370 was marked by red. (B), (C) and (D) Volcano plots presenting the differently expressed miRNAs from GSE34645, GSE34644 and GSE34646. Both mmu-miR-370 and mmu-miR-197 were indicated by blue arrow. **Figure S5.** Involvement of TGFβR2 in FOXO signaling pathway.

## Data Availability

All data used during the current study available from the corresponding author on reasonable request.

## Abbreviations

AUC: Area under ROC curve
CAD: Coronary artery disease
ceRNA: Competing endogenous RNA
circRNAs: Circular RNAs
DM: Diabetes mellitus
ECs: Endothelial cells
EVs: Extracellular vesicles
FDR: False discovery rate
FISH: Fluorescence in situ hybridization
GEO: Gene Expression Omnibus
GO: Gene Ontology
GSEA: Gene set enrichment analysis
HAECs: Human aorta endothelial cells
HDL-C: High-density lipoprotein cholesterol
HUVEC: Human umbilical vein endothelial cell
KEGG: Kyoto Encyclopedia of Genes and Genomes
LDL-C: Low-density lipoprotein cholesterol
ncRNAs: Non-coding RNAs
NTA: Nanoparticle tracking analysis
OE: Overexpresson
PBS: Phosphate buffered saline
PPP: Platelet-poor plasma
qRT-PCR: Quantitative real-time PCR
RBP: RNA-binding protein
RIP: RNA immunoprecipitation
ROC: Receiver operating characteristic
SD: Standard deviation
TC: Total cholesterol
TG: Triglyceride
TIA: Transient ischemic attack
UTR: 3′ Untranslated region
VSMC: Vascular smooth muscle cell
